The article "Clinical Application Effect of Cluster Management in Noninvasive Ventilator Nursing Care of Patients with Severe Heart Failure" was retracted in 2023. Reasons: unreliable results or conclusions; concerns about the data; concerns about the peer review; concerns about the citations.

# Clinical Application Effect of Cluster Management in Noninvasive Ventilator Nursing Care of Patients with Severe Heart Failure

**DOI:** 10.1155/2022/9628213

**Published:** 2022-06-29

**Authors:** Huanli Luo, Guangyu Zhu

**Affiliations:** ^1^Department of Nursing, Henan Vocational College of Nursing, Anyang City, 455000 Henan Province, China; ^2^Four Departments of Cardiovascular Disease Center, Fifth Affiliated Hospital of Sun Yat-Sen University, Zhuhai City, 519000 Guangdong Province, China

## Abstract

**Objective:**

To elucidate the clinical application effect of cluster management in noninvasive ventilator nursing care of patients with severe heart failure (HF).

**Methods:**

A total of 116 severe patients with HF who received treatment in the our hospital between October 2018 and December 2019 were included, including 50 cases (control group) treated with routine nursing and 66 cases (research group) treated with cluster management. The treatment-related indexes (mechanical ventilation time and hospitalization expenses), symptom resolution (dyspnea, insomnia, nausea, and upper abdominal pain), systolic/diastolic blood pressure (SBP/DBP), heart rate (HR), and prognosis (mortality and disability rate) were observed and compared between the two groups.

**Results:**

Statistically shorter time of mechanical ventilation and symptom (dyspnea, insomnia, nausea, and upper abdominal pain) resolution were found in the research group compared with the control group. In addition, the research group showed significantly lower hospitalization expenses, SBP, DBP, and HR than the control group. Moreover, lower mortality and disability rates were determined in the research group, yet with no statistical significance between the two cohorts.

**Conclusion:**

The above results indicate the remarkable clinical application effect of cluster management in noninvasive ventilator nursing of severe HF, which can enhance the treatment efficacy, blood pressure and HR of patients, and facilitate their recovery.

## 1. Introduction

Heart failure (HF) is a common cardiovascular disease that has a great impact on public health, with high medical costs, morbidity, and mortality [1, 2]. According to the statistics of HF, the disease has affected 26 million cases, with the post-diagnosis 1-year and 5-year mortality rates as high as 45% and 60%, respectively [3]. The pathological mechanism of HF is complicated, with pathogenic factors involving hypertension, aging, diabetes, coronary heart disease and obesity, and the major clinical presentations of dyspnea and lower limb edema [4, 5]. Severe HF is mainly characterized by severe symptoms induced by abnormal heart structure and function, which is common in the elderly, especially among elderly women [6]. At present, patients with severe HF can be relieved through noninvasive ventilator intervention. However, most of these elderly patients are unable to take care of themselves independently, nor can they get close care from their families as they are treated in the intensive care unit [7], which puts forward demands for noninvasive ventilator nursing of severe HF. Therefore, related research in this field is of positive significance for improving the curative effect and prognosis of such patients.

HF management interventions are constantly being updated, which also lead to a better understanding of the economic or social burden of HF, thus providing more refined interventions for the treatment of this patient population [8]. Nursing is one of the indispensable management means, which can provide a certain degree of care for hospitalized patients and help them recover and discharge smoothly [9]. Given that severe HF patients have considerable difficulties in self-care, conventional management models may be difficult to meet their rehabilitation needs [10]. Cluster management, on the other hand, is a holistic management intervention method for critically ill patients, which uses multidisciplinary and evidence-based thinking to formulate nursing strategies [11]. It is put forward by the American Institute of Health Promotion, which develops a series of practical and targeted nursing measures to clinical patients according to specific nursing scenarios, with the main goal of improving nursing quality [12, 13]. Currently, cluster management has been widely used in various medical scenarios such as hip fractures, sepsis, and chronic obstructive pulmonary disease, which has a significant positive impact on improving treatment compliance and reducing patient readmission rate [14–16]. In addition, cluster management is effective in the treatment of patients with acute respiratory distress syndrome complicated with ventilator-associated pneumonia, which can not only inhibit the inflammatory response of patients, but also effectively improve lung function [17]. It has also been shown to exert a positive effect on early mobility of patients with mechanical ventilation and can promote the recovery of patients with outstanding safety [18].

Given the current lack of research on the application of cluster management in HF, this study explored the clinical effect of cluster management in noninvasive ventilator nursing of severe HF, aiming to provide new ideas for the management of severe HF patients.

## 2. Materials and Methods

### 2.1. General Information

The study has been approved by the Ethics Committee of the hospital. The study enrolled 116 patients with severe HF who were treated in our hospital between October 2018 and December 2019 and assigned them into the following two groups according to different nursing methods: a control group (*n* = 50) treated with routine nursing and a research group (*n* = 66) intervened by cluster management. The mean age and the male-to-female ratio of the control group were 64.35 ± 9.96 years and 18 : 32 females, respectively, with 33 cases of New York Heart Association (NYHA) grade II, and 17 cases of grade III. In the research group, the mean age and the male-to-female ratio were 66.85 ± 12.88 years and 22 : 44, respectively, with 40 cases of NYHA grade II and 26 cases of NYHA grade III. The two groups were comparable in baseline data with no statistical significance (*P* > 0.05; Table 1).

### 2.2. Inclusion and Exclusion Criteria

Inclusion criteria was as follows: confirmed diagnosis of severe HF; NYHA [19] grades II-III; high patient compliance; use of noninvasive ventilation (NIV); no use of medications that might affect the results of the study in the last six months; normal communication and cognitive function; and signed informed consent provided.

Exclusion criteria was as follows: severe organ dysfunction; malignant tumor(s); infectious diseases or systemic disorders; mental disorders or cognitive impairment; and pregnant or lactating patients.

### 2.3. Interventions

The control group received routine nursing. Patients were given nasal feeding in the conventional supine position and kept a semi-reclining (sitting) position or having the head of the bed elevated 30-45° for 30 minutes. In addition, atomization inhalation was performed twice a day as prescribed. Weaning care and electric sputum aspiration were also provided. Patients were given liquid or semi-liquid food and oral care twice daily with normal saline.

Cluster management was implemented in the research group on the basis of the control group. (1) After communicating with the doctor in charge, the nursing staff raised the head of the bed by 30-45° or placed the patient in a semi-sitting position when the condition allowed. The tail of the bed was also appropriately raised to prevent back skin abrasions caused by body sliding. (2) The atomization device was installed on the patient's ventilator to further strengthen the humidification and warming of the artificial airway. In addition, the humidifier was checked to ensure that the water temperature was 32-35 °C and the gas humidity was 60-70%. The sterile water for injection of the humidifier was replaced once daily, and the regulations that the nebulizer should be replaced and disinfected once a day and special use by special personnel were strictly followed. (3) According to the doctor's advice, patients with stable cardiopulmonary function tried to stop taking sedatives and weaned off every morning. If the patient was successfully weaned, he or she was given a mask to breathe on his or her own. If not, sedatives were re-administered, and face mask ventilators were used, until another try the next day. (4) For patients with NIV, wake-up expectoration was mainly adopted. Nursing staff woke up the patient when turning the patient over and encouraged the patient to cough up sputum after deep inhalation through hollow palm tapping and back shaking, so as to avoid electric sputum suction as much as possible. Sputum aspiration was carried out if the patient was unable to cough, and electrocardiographic monitoring shows increased heart rate (HR) and decreased oxygen saturation. (5) Patients were given oral care twice a day with 5% dilute iodophor solution. In terms of diet, they were fed with small-bore feeding tubes four times a day, each time not exceeding 200 mL.

### 2.4. Outcome Measures

The treatment of patients, which was mainly assessed from the following parameters, was observed and compared between the two groups: (1) The mechanical ventilation time and hospitalization cost were recorded; (2) symptom improvement was evaluated by recording the resolution time of symptoms such as dyspnea, insomnia, nausea, and upper abdominal pain; (3) the systolic blood pressure (SBP), diastolic blood pressure (DBP), and HR were recorded before and after intervention; and (4) patients' outcomes were assessed by recording mortality and disability rates during care.

### 2.5. Statistical Methods

Data processing and image export were made by SPSS *v*17.0 (IBM Corp., Armonk, NY, USA) and GraphPad Prism *v*6 (GraphPad Software, Inc., San Diego, CA, USA), respectively. The categorical data were recorded in the form of number of cases/percentages (n/%), and intergroup comparisons of data such as age, NYHA classification, hypertensive heart disease, coronary heart disease, and dilated cardiomyopathy in Table 1 were performed by the *χ*2 test. Quantitative data were denoted by mean ± SD, and independent samples *t*-test was used to compare data between groups (such as mechanical ventilation time and hospitalization cost in Figure 1 and improvement time of dyspnea, insomnia, nausea, and upper abdominal pain Figure 2), while paired *t*-test was used for intragroup comparisons before and after intervention (such as SBP, DBP, and HR in Figure 3). Differences with *P* < 0.05 were considered statistically significant.

## 3. Results

### 3.1. The General Data of the Two Groups Are Comparable

The control group and the research group showed no significant differences in general data such as age, mean age, sex, course of disease, NYHA classification, hypertensive heart disease, coronary heart disease, dilated cardiomyopathy, and family history of HF (*P* > 0.05; Table 1).

### 3.2. Cluster Management Improves the Treatment of Severe HF Patients

We evaluated the effects of the two interventions on patients with severe HF by comparing the duration of mechanical ventilation and hospitalization costs. The data showed that the time of mechanical ventilation was shorter and the hospitalization cost was lower in the research group compared with the control group, with statistical significance (*P* < 0.05; Figure 1).

### 3.3. Cluster Management Improves Symptoms in Patients with Severe HF

We compared the symptom (dyspnea, insomnia, nausea, and upper abdominal pain) resolution time between the two groups to analyze the effects of the two interventions on symptom improvement. Statistically, the resolution time of the above symptoms was lower in the research group compared with the control group (*P* < 0.05; Figure 2).

### 3.4. Cluster Management Improves Blood Pressure (BP) and HR in Patients with Severe HF

We measured the BP and HR of the two cohorts of patients. The data showed no significant difference in SBP, DBP, and HR between the two groups before intervention (*P* > 0.05). After intervention, SBP, DBP, and HR reduced significantly in both groups (*P* < 0.05), and their levels in the research group were significantly lower than those in the control group (*P* < 0.05; Figure 3).

### 3.5. Cluster Management Improves the Prognosis of Severe HF Patients

We evaluated the prognostic impact of the two interventions on patients with severe HF by recording the mortality and disability rates during nursing care. The results determined lower mortality and disability rates in the research group compared with the control group, but with no statistical significance (*P* > 0.05, Figure 4).

## 4. Discussion

HF, a progressive disease with complex pathological mechanisms, is related to ventricular filling (diastole) or blood ejection (systole) damage, which leads to weakness, shortness of breath, dyskinesia, and other symptoms of insufficient blood supply [20]. The effectiveness of NIV has been demonstrated in patients with acute respiratory failure, which can not only improve patient prognosis, but also reduce the need for invasive mechanical ventilation [21, 22]. While in addition to NIV, effective management intervention in patients with severe HF may exert beneficial effects on improving treatment efficacy, symptoms and patient prognosis.

More and more researchers have analyzed the intervention effects of different management models on HF patients. For example, Zhou et al. [23] pointed out that while validly mitigating negative emotions, evidence-based nursing can improve the quality of life and long-term curative effect of patients with acute myocardial infarction complicated with HF. Guan et al. [24] reported that the application of integrated healthcare intervention in patients with acute HF can significantly enhance the quality of care and promote the recovery of patients' physical function. And Zhao et al. [25] showed in their meta-analysis that self-management interventions can significantly improve disease-related cognition and quality of life of HF patients and reduce HF-related hospitalization costs. In this study, we gave routine nursing intervention to patients in the control group, mainly including basic nursing in lying position, diet, weaning, atomization therapy, sputum aspiration, and oral hygiene. For those in the research group, cluster management, with similar nursing contents but more elaborate nursing measures and higher requirements for nursing staff, was added on the basis of routine nursing. Our data revealed significantly less mechanical ventilation time and hospitalization cost of the research group under cluster management, which is consistent with the research results of Shi et al. [26]. It suggests that cluster management can improve the treatment of severe HF patients at a lower cost, which may also be related to shorter duration of mechanical ventilation. Besides, the research group outperformed the control group in the improvement of symptoms, which is manifested as faster resolution of dyspnea, insomnia, nausea, upper abdominal pain and other symptoms. In terms of BP and HR, cluster management also shows more favorable advantages, with more significant improvement in patients' SBP, DBP, and HR than the conventional care. Finally, we analyzed the prognosis of patients in both groups. The mortality and disability rate of patients with cluster management were found to be lower, but with no statistical significance compared with the control group, suggesting that cluster management had the same improvement effect on the prognosis of patients with severe HF as routine nursing. Instead of giving conventional electric sputum aspiration and weaning care directly, patients in the research group were encouraged to do spontaneous expectoration according to their specific conditions in the process of cluster management and were given electric sputum aspiration only when spontaneous expectoration was ineffective, which can prevent airway injury and lung infection caused by frequent sputum aspiration [27]. At the same time, the weaning adaptation training further exercises patients' weaning adaptation ability, which is of positive significance for improving patients' symptoms and signs, shortening hospitalization time, and even reducing hospitalization costs. Andryukhin et al. [28] pointed out in their study that cluster management not only significantly improved the emotional state and quality of life of HF patients, but also had positive effects on their walking ability, cardiac function, and lipid status.

The novelty of this study lies in the multidimensional analysis of the application of cluster management in severe HF patients from treatment conditions such as mechanical ventilation time and hospitalization cost; improvement of symptoms such as dyspnea, insomnia, nausea, and upper abdominal pain; BP and HR; and patient prognosis such as mortality and disability rate, which confirms the effectiveness, reliability, and safety of this care model in noninvasive ventilator nursing of patients with severe HF, providing clinical research for the management optimization of such patients. However, there are still some deficiencies in this study. First, the sample size of this study is small, and the accuracy of the experimental results will be further improved if a multicenter study with more samples can be carried out. Second, this study did not analyze the long-term outcomes of patients, which could be supplemented to further understand the impacts of different management models on patients' long-term outcomes. Finally, supplementary analysis of risk factors affecting the prognosis of severe HF patients from the aspect of nursing measures will be beneficial to further improve the quality of nursing.

## 5. Conclusion

To sum up, this study proposes for the first time that cluster management has a promising clinical application prospect in noninvasive ventilator nursing of patients with severe HF, as it can not only shorten mechanical ventilation time, reduce hospitalization expenses, but also significantly improve the symptoms and signs of patients.

## Figures and Tables

**Figure 1:** Treatment of two groups of patients. (a) Mechanical ventilation time of patients in the two groups. (b) Hospitalization expenses of patients in the two groups. Note: ∗∗*P* < 0.01. The data between groups were analyzed by the independent samples *t* test.

**Figure 2:** Symptom improvement of two groups of patients. (a) Resolution time of dyspnea in two groups. (b) Resolution time of insomnia in two groups. (c) Resolution time of nausea in two groups. (d) Resolution time of upper abdominal pain in two groups. Note: ∗∗*P* < 0.01. The data between groups were analyzed by the independent samples *t* test.

**Figure 3:** Blood pressure and heart rate of patients in two groups. (a) SBP of patients in two groups. (b) DBP of patients in two groups. (c) HR of patients in two groups. Note: ∗*P* < 0.05; ∗∗*P* < 0.01. The data before and after intervention were analyzed by the paired *t*-test.

**Figure 4:** Patient outcomes in two groups. (a). Case fatality rate of patients in two groups. (b). Disability rate of patients in two groups. Note: The data between groups were analyzed by the Chi-square test.

**Table 1:** Baseline data of patients in the two groups (*n* (%), mean ± SD).

Factors	*n*	Control group (*n* = 50)	Research group (*n* = 66)	*χ* 2/t	*P*
Age (years)				0.181	0.671
<65	49	20 (40.00)	29 (43.94)		
≥65	67	30 (60.00)	37 (56.06)		
Average age (years)	116	64.35 ± 9.96	66.85 ± 12.88	1.138	0.257
Gender				0.090	0.765
Male	40	18 (36.00)	22 (33.33)		
Female	76	32 (64.00)	44 (66.67)		
Course of disease (years)	116	4.68 ± 1.22	4.50 ± 1.20	0.794	0.429
NYHA classification				0.355	0.551
II	73	33 (66.00)	40 (60.61)		
III	43	17 (34.00)	26 (39.39)		
Hypertensive heart disease				0.014	0.906
Without	68	29 (58.00)	39 (59.09)		
With	48	21 (42.00)	27 (40.91)		
Coronary heart disease				0.105	0.746
Without	56	25 (50.00)	31 (46.97)		
With	60	25 (50.00)	35 (53.03)		
Dilated cardiomyopathy				0.225	0.635
Without	105	46 (92.00)	59 (89.39)		
With	11	4 (8.00)	7 (10.61)		
Family history of heart failure				0.166	0.683
Without	88	37 (74.00)	51 (77.27)		
With	28	13 (26.00)	15 (22.73)		

## Data Availability

The simulation experiment data used to support the findings of this study are available from the corresponding author upon request.
